This article has been retracted.

# Analysis of Clinical Effects of Comprehensive Nursing Based on Enhanced Recovery after Surgery in Patients with Embolization for Intracranial Aneurysms

**DOI:** 10.1155/2022/3026680

**Published:** 2022-07-08

**Authors:** Jing Liu, Kunxian Zhang, Bei Wang, Qin Hu, Qing Zhang, Lei Wan, Xianpu Wang, Wenping Xiong

**Affiliations:** ^1^Department of Anesthesia, Zhongnan Hospital of Wuhan University, Wuhan, 430071 Hubei, China; ^2^Department of Neurosurgery, Zhongnan Hospital of Wuhan University, Wuhan, 430071 Hubei, China

## Abstract

**Objective:**

This research sets out to elucidate the clinical effect of comprehensive nursing based on the concept of enhanced recovery after surgery (ERAS) in patients with embolization for intracranial aneurysms (IAs).

**Methods:**

This study enrolled 119 patients with embolization for IAs in the Zhongnan Hospital of Wuhan University from January 2020 to January 2021 and divided them into two groups according to the perioperative care they received: a control group (*n* = 39) treated with routine perioperative nursing and an observation group (*n* = 80) treated with ERAS-based comprehensive nursing. Surgical indicators, neurological function (National Institute of Health Stroke Scale (NIHSS) score; Scandinavian Stroke Scale (SSS) score), anxiety and depression (Self-Rating Anxiety Scale (SAS) score; Self-Rating Depression Scale (SDS) score), incidence of adverse events, and patient satisfaction were compared.

**Results:**

The observation group had better surgical indicators and lower scores of NIHSS, SSS, SAS, and SDS than the control group, accompanied by a lower incidence of adverse events and higher patient satisfaction.

**Conclusions:**

ERAS-based comprehensive nursing can better promote patients' neurological recovery after embolization for IAs, relieve unhealthy emotions (depression, anxiety, etc.), and reduce the occurrence of adverse reactions, facilitating patient discharge.

## 1. Introduction

Intracranial aneurysm (IA) is a common, devastating condition that can lead to death or permanent disability, affecting approximately 2-5% of the general population [1, 2]. Such a tumor is often found by accident during brain examinations and other procedures. If ruptured, it is very easy to cause subarachnoid hemorrhage (SAH), which is the reason for the high morbidity and mortality of IAs [3]. IA-induced SAH not only contributes to a mortality rate as high as 20% but also a high recurrence rate in surviving patients [4]. Age, sex, hypertension, aneurysm size, and smoking have long been identified as risk factors [5]. However, the etiology of SAH, especially the rupture risk of IAs, has not been completely elucidated and needs further research [6]. In recent years, the research on the treatment plan and outcome of SAH caused by IAs has become the main research direction [7, 8]. Exploring effective intervention models for IAs is of great practical significance for further optimizing the management of such patients and improving their prognosis.

IAs are routinely treated by endovascular therapy [9, 10], among which the most extensively used is coil embolization (CE), with the common strategies being routine CE, balloon-assisted CE, and stent-assisted CE [11]. Despite its wide application, the use of CE is often associated with a high recurrence rate, especially in the treatment of large and giant IAs [12]. And although stent-assisted CE can help achieve a more lasting curative effect, the postoperative recurrence rate of IAs can be as high as 20-57% in the patients treated [13, 14]. Hence, further and effective postoperative care is required, which can significantly improve the effectiveness of treatment and ensure the safety of patients during treatment [15]. Among them, comprehensive nursing is a brand-new nursing model integrating the advantages of group nursing and primary nursing, which is a perfect combination of nursing concept, nursing plan, and nursing quality evaluation [16]. The purpose of this study is to explore the clinical effect of comprehensive nursing based on the concept of enhanced recovery after surgery (ERAS) on patients with embolization for IAs.

## 2. Methods

### 2.1. General Information

This study enrolled 119 cases of IAs undergoing embolization in the Neurosurgery Department of Zhongnan Hospital of Wuhan University from January 2020 to January 2021. All patients were diagnosed as IA by computed tomography angiography (CTA) examination and met the inclusion criteria. All cases underwent CE or stent-assisted CE for IAs. Patients were divided into either the control group (CG; *n* = 39), which received routine perioperative care after IA embolization, or the observation group (OG; *n* = 80), which received perioperative comprehensive nursing based on the concept of enhanced recovery after surgery (ERAS). The two cohorts were similar in sex, age, and course of disease, with comparability (*P* > 0.05). Inclusion criteria are as follows: patients who can accurately express their discomfort and met the indications of interventional embolization with Hunt-Hess grade 0-2 IAs were included [17]. Exclusion criteria are as follows: patients with underlying medical conditions, surgical contraindications, or other types of nervous system diseases (hypertensive cerebral hemorrhage, craniocerebral trauma, etc.) were excluded.

The patients' family members agreed to this study and signed the relevant agreement, and this study has obtained ethical approval from the Zhongnan Hospital of Wuhan University.

### 2.2. Methods

CG received routine nursing, including closely monitoring patients' vital signs after operation, answering questions raised by patients and their families in detail, reminding patients' families of matters needing attention during the implementation of care for patients, maintaining the sanitary environment of the ward, and paying strict attention to disinfection procedures. On the basis of the above measures, OG was given ERAS-based comprehensive rehabilitation nursing. First of all, patients were provided with psychological care. Patients' negative emotions (NEs) were evaluated and divided into three grades: no NE, certain NEs, and severe NEs. For those who had no NEs, their family members were reminded to pay attention to observation; for those with certain NEs, psychological counseling and comfort were given, and methods such as attention diversion, suggestion, and encouragement were combined to help them relieve. For those with severe NEs, individualized counseling was provided, family members were reminded to give emotional support, and professional psychiatric medical staff were invited for intervention. At the same time, rehabilitation health education was carried out for patients. The postoperative situation of each patient was investigated and statistically analyzed to understand his/her needs for rehabilitation-related health education and knowledge points. Besides, family members were given supporting health knowledge guidance, including information about the operation effect, rehabilitation plan at different stages after operation, postoperative dietary and activity precautions, approximate hospitalization time, and precautions after discharge. In case of adverse events (AEs), patients were informed in detail about prevention and control and were instructed to understand the common causes of postoperative AEs and prevention techniques. Patients with transient neurological dysfunction were given slow intravenous injection of nimetone with micropump immediately. Those at high risk of cerebral vasospasm were given oral intervention of nimodipine tablets. In addition, patients were closely observed for neurological symptoms, such as muscle strength decline, dizziness, nausea, and vomiting. And the nursing staff would immediately report to the attending doctor and coordinate the emergency treatment for the patient if the above neurological symptoms occurred. Furthermore, the patient's blood pressure was continuously monitored. For those whose blood pressure increased continuously or suddenly, the risk of rebleeding was assumed to be higher, and immediate antihypertensive measures were taken to maintain the mean arterial pressure of 10 to 11 kPa. Bleeding at the puncture site and subcutaneous hematoma are also major AEs that affect postoperative recovery. In such cases, the puncture site was bandaged after compression with sandbags, and the patient was reminded to lie supine without a pillow.

### 2.3. Endpoints

#### 2.3.1. Surgical Indicators

The surgical indicators (early ambulation and length of stay (LOS)) of patients were compared.

#### 2.3.2. Neurological Function

Patients' neurological function assessed by the National Institute of Health Stroke Scale (NIHSS; score range: 0-42 points) [18] and Scandinavian Stroke Scale (SSS; score range: 0-58 points) [19] was compared between groups. The better the patient's neurological function, the lower the score.

#### 2.3.3. Mental Health (MH)

Patients' MH before and 1 month after nursing, evaluated using the Self-Rating Anxiety/Depression Scale (SAS/SDS) (20 items, 0-100 points) [20, 21], was also observed and compared. The worse the MH level of patients, the higher the scores.

#### 2.3.4. Incidence of AEs

The two groups were also compared in terms of the incidence of AEs (cerebral vasospasm, rebleeding, headache, vomiting, bleeding at the puncture site, and subcutaneous hematoma).

#### 2.3.5. Patient Satisfaction

The nursing satisfaction, assessed using the self-made nursing satisfaction questionnaire with self-designed contents and evaluation criteria, was compared between groups. The total score is 100 points, of which 100-85 is considered as satisfactory, 60-84 as basically satisfactory, and less than 60 as dissatisfied. Satisfaction = (satisfied + basically satisfied) cases/total cases∗100%.

### 2.4. Statistical Processing

SPSS22.0 (AsiaAnalytics formerly SPSS China) was employed for comprehensive data analysis and GraphPad Prism 6 (GraphPad Software, San Diego, USA) for graph drawing. The statistical methods for the comparison of measurement data expressed as *X* ± *S* were *t*-test (intergroup) and paired *t*-test (within-group before and after intervention), while counting data represented by number of cases/percentage (*n*/%) were analyzed by the *χ*^2^. The significance level was assumed at *P* < 0.05.

## 3. Results

### 3.1. General Information

The two cohorts showed no statistical differences in a series of general data like gender, age, and average income (*P* > 0.05; Table 1).

### 3.2. Surgical Indicators

The comparison of the postoperative indicators determined earlier ambulation and shorter LOS in OG versus CG, with statistical significance (*P* < 0.05; Figure 1).

### 3.3. Neurological Function

The comparison of NIHSS and SSS scores showed that the two scores decreased obviously at 1 month after care, especially in OG (*P* < 0.05; Figure 2).

### 3.4. MH

After comparing SAS and SDS scores, it was found that the two scores dropped statistically after care in both groups and were lower in OG (*P* < 0.05; Figure 3).

### 3.5. Incidence of AEs

After investigating the incidence of AEs in the two groups, it was found that the incidence was significantly lower in OG compared with CG (*P* < 0.05; Table 2).

### 3.6. Patient Satisfaction

OG was far superior to CG in patient satisfaction, as indicated by the patient satisfaction survey (*P* < 0.05; Table 3).

## 4. Discussion

After surgery for IAs, a few patients may still experience IA recurrence [7]. In addition, aneurysm rupture that is prone to during surgery significantly increases the risk of morbidity and mortality [22]. Therefore, reasonable nursing methods are needed to delay aneurysm rupture and slow down postoperative aneurysm recurrence [23, 24]. In this section, we will combine the research results to discuss the role of ERAS-based comprehensive nursing on patients' postoperative recovery.

From the perspective of neurological function, the NIHSS and SSS scores in OG using ERAS-based comprehensive nursing were significantly lower compared with CG, indicating that ERAS-based comprehensive nursing improved the neurological function of patients postoperatively. In addition to high mortality and recurrence rates, ruptured aneurysms and subsequent intracranial hemorrhage leave most survivors with severe neurological deficits [25]. Ruptured aneurysms may cause intracranial artery injury, which will lead to increased oxidative stress and massive inflammatory reactions that will further aggravate the pathological changes of intracranial artery wall, thus affecting the nervous system [26, 27]. Therefore, many clinical studies focus not only on rupture prevention and prophylactic therapy during treatment but also postoperative nursing intervention, which focuses on those aneurysms that are at risk of rupture. However, the current nursing intervention for these aneurysms remains a huge challenge [28]. Among various nursing methods, comprehensive nursing intervention has the advantages of strong pertinence and wide coverage, which contributes to a better nursing intervention effect on patients and a good relationship between patients and medical staff. Besides, it provides better health education, medical care and other interventions that enable patients to actively participate in the treatment, with higher medication compliance and satisfaction, leading to positive treatment outcomes and faster patient recovery [29]. Compared with comprehensive nursing, conventional nursing mode is inferior in medication, health care, and the establishment of doctor-patient relationship, and it is impossible to care for patients in all aspects [30]. Therefore, patients in OG recovered faster in terms of neurological recovery due to better postoperative care and better targeted medication care after surgery. Li et al. [31] also demonstrated beneficial effects of ERAS-based comprehensive nursing on the neurological function of patients with knee osteoarthritis after total knee arthroplasty, which is similar to our study.

In addition to impaired limb function of patients at all levels, neurological damage has a great impact on patients' gastrointestinal function, resulting in a great decline in patients' quality of life and difficulty in recovery [32, 33]. Combing the detection results of two surgical indicators in this study, OG using ERAS-based comprehensive nursing not only had earlier ambulation but also faster discharge, with fewer postoperative AEs. Similarly, Lv et al. [34] pointed out in their study that ERAS-based comprehensive nursing not only significantly promoted postoperative rehabilitation of patients with craniocerebral trauma but also reduced the incidence of postoperative complications. This study also found faster and more efficient elimination of psychological anxiety and depression in OG. Xie et al. [35] reported that the NEs of patients with cerebral infarction were significantly alleviated after ERAS combined with continuous nursing, which is consistent with our findings. In the recovery of various diseases, NEs will not only weaken the recovery effect of patients but also aggravate their illness. Among neurological diseases, unhealthy psychological emotions are closely linked to an increased risk. And effective intervention will not only reduce the damaged nervous system function but also mitigate depression, so that they can get out of the vicious circle [36, 37]. On the whole, because of the implementation of more targeted comprehensive nursing for patients in OG based on ERAS, the treatment effect of patients was better, and the nervous system was better recovered, so that patients could ambulate earlier with effective relief of psychological anxiety and depression. This also enables patients to better cooperate with the treatment, with fewer AEs and faster discharge. A similar study found that in perioperative care of patients with IAs, comprehensive nursing can shorten the LOS of patients, reduce complications and infections, and improve patient satisfaction [38], similar to our findings.

The novelty of this study is that it confirms the effectiveness, reliability, and safety of ERAS-based comprehensive nursing in the clinical application of IAs in terms of surgical indications, neurological function, MH, incidence of adverse reactions, and patient satisfaction, providing a new option for the management optimization of IA patients. However, some shortcomings of this study need to be addressed. First, some related indicators and inflammatory factors have not been measured. Besides, patient compliance during treatment is also worthy of investigation. In the future research, we will further test related factors while constantly improving the treatment and nursing programs to better benefit patients.

To sum up, the application of comprehensive nursing based on ERAS concept can promote the neurological recovery of patients with embolization for IAs; reduce depression, anxiety, and AEs in patients; and enable patients to be discharged faster, which is worth popularizing in clinic.

## Figures and Tables

**Figure 1:** Surgical indicators. (a) Time for ambulation: the time of ambulation was faster in the observation group than in the control group (*P* < 0.05). (b) Length of stay: the length of stay was shorter in the observation group compared with the control group (*P* < 0.05). Note: ^∗^*P* < 0.05 vs. control group.

**Figure 2:** Neurological function of patients in the two groups. (a) NIHSS score: after nursing for one month, the NIHSS score was significantly lower in the observation group compared with the control group (*P* < 0.05). (b) SSS score: after one month of nursing, the SSS score was significantly lower in the observation group than in the control group (*P* < 0.05). Note: ^∗^*P* < 0.05 vs. before nursing; #*P* < 0.05 vs. control group.

**Figure 3:** Mental health of patients in two groups. (a) SAS score: the SAS score of the two groups changed significantly after one month of nursing and was lower in the observation group compared with the control group (*P* < 0.05). (b) SDS score: the SDS score of the two groups changed significantly after one month of nursing and was lower in the observation group compared with the control group (*P* < 0.05). Note: ^∗^*P* < 0.05 vs. before nursing; #*P* < 0.05 vs. control group.

**Table 1:** General information of patients in the two groups.

Classification	Observation group (*n* = 80)	Control group (*n* = 39)	*t*/*χ*^2^	*P*
Sex			0.150	0.698
Male	42 (52.50)	19 (48.72)		
Female	38 (47.50)	20 (51.28)		
Age (years old)	52.88 ± 7.68	53.28 ± 7.82	0.265	0.791
BMI (kg/m^2^)	23.17 ± 2.68	23.26 ± 2.39	0.178	0.859
Residence			0.053	0.819
Urban	60 (75.00)	30 (76.92)		
Rural	20 (25.00)	9 (23.08)		
Eating habits			0.261	0.609
Light	23 (28.75)	13 (33.33)		
Heavy	57 (71.25)	26 (66.67)		
Smoking			1.006	0.316
Yes	64 (80.00)	28 (71.79)		
No	16 (20.00)	11 (28.21)		
Drinking			0.136	0.712
Yes	56 (70.00)	26 (66.67)		
No	24 (30.00)	13 (33.33)		

**Table 2:** Incidence of adverse events in the two groups.

Classification	Observation group (*n* = 80)	Control group (*n* = 39)	*χ* ^2^	*P*
Cerebral vasospasm	0 (0.00)	2 (5.13)	—	—
Rebleeding	0 (0.00)	1 (2.56)	—	—
Headache	0 (0.00)	0 (0.00)	—	—
Vomiting	1 (1.25)	1 (2.56)	—	—
Bleeding at the puncture site	0 (0.00)	1 (2.56)	—	—
Subcutaneous hematoma	1 (1.25)	1 (2.56)	—	—
Incidence of adverse events (%)	2 (2.50)	6 (15.38)	6.941	0.008

**Table 3:** Satisfaction of two groups of patients.

Classification	Observation group (*n* = 80)	Control group (*n* = 39)	*χ* ^2^	*P*
Satisfied	56 (70.00)	19 (48.72)	—	—
Basically satisfied	20 (25.00)	11 (28.21)	—	—
Dissatisfied	4 (5.00)	9 (23.07)	—	—
Satisfaction (%)	76 (95.00)	30 (76.93)	8.804	0.003

## Data Availability

The labeled dataset used to support the findings of this study are available from the corresponding author upon request.

## References

[1] Shimizu K., Kataoka H., Imai H. (2021). Hemodynamic force as a potential regulator of inflammation-mediated focal growth of saccular aneurysms in a rat model. *Journal of Neuropathology and Experimental Neurology*.

[2] Xu Z., Rui Y. N., Hagan J. P., Kim D. H. (2019). Intracranial aneurysms: pathology, genetics, and molecular mechanisms. *Neuromolecular Medicine*.

[3] Etminan N., Dorfler A., Steinmetz H. (2020). Unruptured intracranial aneurysms- pathogenesis and individualized management. *Deutsches Ärzteblatt International*.

[4] Samuels O. B., Sadan O., Feng C. (2021). Aneurysmal subarachnoid hemorrhage: trends, outcomes, and predictions from a 15-year perspective of a single neurocritical care unit. *Neurosurgery*.

[5] Hamdan A., Barnes J., Mitchell P. (2014). Subarachnoid hemorrhage and the female sex: analysis of risk factors, aneurysm characteristics, and outcomes. *Journal of Neurosurgery*.

[6] Greving J. P., Wermer M. J., Brown R. D. (2014). Development of the phases score for prediction of risk of rupture of intracranial aneurysms: a pooled analysis of six prospective cohort studies. *Lancet Neurology*.

[7] Lovik K., Laupsa-Borge J., Logallo N., Helland C. A. (2021). Dyslipidemia and rupture risk of intracranial aneurysms-a systematic review. *Neurosurgical Review*.

[8] Zhou G., Zhu Y. Q., Su M., Gao K. D., Li M. H. (2016). Flow-diverting devices versus coil embolization for intracranial aneurysms: a systematic literature review and meta-analysis. *World Neurosurgery*.

[9] McDonald J. S., McDonald R. J., Fan J., Kallmes D. F., Lanzino G., Cloft H. J. (2013). Comparative effectiveness of unruptured cerebral aneurysm therapies: propensity score analysis of clipping versus coiling. *Stroke*.

[10] Lin N., Cahill K. S., Frerichs K. U., Friedlander R. M., Claus E. B. (2018). Treatment of ruptured and unruptured cerebral aneurysms in the USA: a paradigm shift. *Journal of Neurointerventional Surgery*.

[11] Xia J. L., Li G. L., Liu H. E., Feng-Fei X., Gu X. D. (2021). Flow-diverting device versus coil embolization for unruptured intracranial aneurysm. *Medicine (Baltimore)*.

[12] Ding Y. H., Ghozy S., Dai D., Brinjikji W., Kallmes D. F., Kadirvel R. (2022). Rabbit elastase aneurysm model mimics the recurrence rate of human intracranial aneurysms following platinum coil embolization. *AJNR. American Journal of Neuroradiology*.

[13] Consoli A., Vignoli C., Renieri L. (2016). Assisted coiling of saccular wide-necked unruptured intracranial aneurysms: stent versus balloon. *Journal of Neurointerventional Surgery*.

[14] Wang B., Gao B. L., Xu G. P., Xiang C., Liu X. S. (2015). Endovascular embolization is applicable for large and giant intracranial aneurysms: experience in one center with long-term angiographic follow-up. *Acta Radiologica*.

[15] Hayes J., Peruzzi P. P., Lawler S. (2014). Micrornas in cancer: biomarkers, functions and therapy. *Trends in Molecular Medicine*.

[16] Gou Y., Yi J., Jiang M., Cao C. (2019). Analysis on effects of comprehensive nursing care applied in interventional therapy for patients with liver cirrhosis and liver cancer. *Iranian Journal of Public Health*.

[17] Bogli S. Y., Wang S., Romaguera N. (2022). Impact of seizures and status epilepticus on outcome in patients with aneurysmal subarachnoid hemorrhage. *Neurocritical Care*.

[18] Eskioglou E., Huchmandzadeh Millotte M., Amiguet M., Michel P. (2018). National Institutes of Health Stroke Scale zero strokes. *Stroke*.

[19] Stubbs P. W., Mortensen J. (2020). Clinimetrics: the Scandinavian stroke scale. *Journal of Physiotherapy*.

[20] Li H., Jin D., Qiao F., Chen J., Gong J. (2016). Relationship between the self-rating anxiety scale score and the success rate of 64-slice computed tomography coronary angiography. *International Journal of Psychiatry in Medicine*.

[21] Jokelainen J., Timonen M., Keinanen-Kiukaanniemi S., Harkonen P., Jurvelin H., Suija K. (2019). Validation of the zung self-rating depression scale (SDS) in older adults. *Scandinavian Journal of Primary Health Care*.

[22] Kocur D., Przybylko N., Bazowski P., Baron J. (2018). Rupture during coiling of intracranial aneurysms: predictors and clinical outcome. *Clinical Neurology and Neurosurgery*.

[23] Lee W. J., Byun J. S., Kim J. K., Nam T. K. (2017). Quantitative computed tomographic volumetry after treatment of a giant intracranial aneurysm with a pipeline embolization device. *Yonsei Medical Journal*.

[24] Wright I. (2007). Cerebral aneurysm--treatment and perioperative nursing care. *AORN Journal*.

[25] Hallikainen J., Keranen S., Savolainen J. (2021). Role of oral pathogens in the pathogenesis of intracranial aneurysm: review of existing evidence and potential mechanisms. *Neurosurgical Review*.

[26] Pascale C. L., Martinez A. N., Carr C. (2020). Treatment with dimethyl fumarate reduces the formation and rupture of intracranial aneurysms: role of Nrf2 activation. *Journal of Cerebral Blood Flow and Metabolism*.

[27] Saqr K. M., Rashad S., Tupin S. (2020). What does computational fluid dynamics tell us about intracranial aneurysms? A meta-analysis and critical review. *Journal of Cerebral Blood Flow and Metabolism*.

[28] Kotowski M., Naggara O., Darsaut T. E. (2013). Safety and occlusion rates of surgical treatment of unruptured intracranial aneurysms: a systematic review and meta-analysis of the literature from 1990 to 2011. *Journal of Neurology, Neurosurgery, and Psychiatry*.

[29] Davis L. L., Fink A. M., Taylor-Piliae R. E. (2019). American heart association council on cardiovascular and stroke nursing liaison report from the development committee. *The Journal of Cardiovascular Nursing*.

[30] Liu J., Xun Z. (2021). Evaluation of the effect of comprehensive nursing in psychotherapy of patients with depression. *Computational and Mathematical Methods in Medicine*.

[31] Li Z., Li B., Wang G. (2021). Impact of enhanced recovery nursing combined with limb training on knee joint function and neurological function after total knee arthroplasty in patients with knee osteoarthritis. *American Journal of Translational Research*.

[32] Bunketorp-Kall L., Pekna M., Pekny M., Samuelsson H., Blomstrand C., Nilsson M. (2020). Motor function in the late phase after stroke: stroke survivors’ perspective. *Annals of Rehabilitation Medicine*.

[33] Du W., Zhao X., Wang Y. (2020). Gastrointestinal bleeding during acute ischaemic stroke hospitalisation increases the risk of stroke recurrence. *Stroke and Vascular Neurology*.

[34] Lv X., Lv F., Yin G., Yi J., Liu Y., Tian Y. (2021). Curative effect of early full nursing combined with postdischarge continuation nursing on patients after craniocerebral trauma. *Evidence-based Complementary and Alternative Medicine*.

[35] Xie R., Chen Y., Chen K., Chen Z. (2021). Intervention effect of rapid rehabilitation nursing combined with continuous nursing after discharge on patients with cerebral infarction in recovery period and the changes in motor function, mental state, and quality of life. *Evidence-based Complementary and Alternative Medicine*.

[36] Wu L., Zhang L. (2017). Effect of high-quality nursing on improvement of anxiety and depression of patients with acute stroke in MRI examination. *Iranian Journal of Public Health*.

[37] Aberg M. A., Toren K., Nilsson M. (2016). Nonpsychotic mental disorders in teenage males and risk of early stroke: a population-based study. *Stroke*.

[38] Xu Y., Wang R. Y., Zhao Y. H. (2021). Effects of perioperative comprehensive nursing based on risk prevention for patients with intracranial aneurysm. *International Journal of Clinical Practice*.

